The article "TAZ promotes cell growth and inhibits Celastrol-induced cell apoptosis" was published in 2016. Journal: Biosci Rep.

# TAZ promotes cell growth and inhibits Celastrol-induced cell apoptosis

**DOI:** 10.1042/BSR20160135

**Published:** 2016-09-29

**Authors:** Shuren Wang, Kai Ma, Lechuang Chen, Hongxia Zhu, Shufang Liang, Mei Liu, Ningzhi Xu

**Affiliations:** * Laboratory of Cell and Molecular Biology & State Key Laboratory of Molecular Oncology, National Cancer Center/Cancer Hospital, Chinese Academy of Medical Sciences and Peking Union Medical College, Beijing 100021, China; † State Key Laboratory of Biotherapy and Cancer Center, West China Hospital, Sichuan University, and Collaborative Innovation Center for Biotherapy, No.17, 3rd Section of People's South Road, Chengdu 610041, P.R. China

**Keywords:** anti-apoptosis, Celastrol, proliferation, transcriptional co-activators with PDZ-binding motif (TAZ)

## Abstract

Hippo pathway is a highly conservative signalling pathway related to the development of organisms, which has been demonstrated to be strongly linked to the tumorigenesis and tumour progression. As the major downstream effector of Hippo pathway, yes-associated protein (YAP), is a transcriptional activator of target genes that are involved in cell proliferation and survival. As an oncogene, YAP can promote cell growth and inhibit cell apoptosis. Another major downstream effector of Hippo pathway, transcriptional co-activators with PDZ-binding motif (TAZ), is nearly 60% homologous with YAP. In the present study, we assume that TAZ probably has the similar function to YAP. To test this issue, we established an inducible and a stable expression system of TAZ in T-Rex-293 and HEK293 cells respectively. The results of cell growth curves, colony formation assay and tumour xenograft growth showed that overexpression of TAZ could promote cell growth *in vitro* and *in vivo*. Meanwhile, we found that up-regulated expression of TAZ could partially restore Celastrol-induced cell apoptosis. Induced overexpression of TAZ could up-regulate its target genes including ankyrin repeat domain-containing protein (ANKRD), cysteine-rich 61 (CYR61) and connective tissue growth factor (CTGF), increase the expression of B-cell lymphoma-2 (Bcl-2), decrease the expression of Bcl-2 associated X protein (Bax) and activate the phosphatidylinositol 3-kinase (PI3K)/protein kinase B (Akt) pathway, which may be the mechanism underlying anti-apoptosis of TAZ. All these findings indicated that TAZ acts as an oncogene that could be a key regulator of cell proliferation and apoptosis.

## Abstract (precis)

TAZ could promote cell proliferation and inhibit Celastrol-induced cell apoptosis. Up-regulation of B-cell lymphoma-2 (Bcl-2), down-regulation of Bcl-2 associated X protein (Bax) and activation of the phosphatidylinositol 3-kinase (PI3K)/protein kinase B (Akt) pathway may be the mechanism underlying anti-apoptosis of TAZ.

The article "TAZ promotes cell growth and inhibits Celastrol-induced cell apoptosis" was published in 2016. Journal: Biosci Rep.

## INTRODUCTION

Hippo pathway, first discovered in *Drosophila*, aims at adjusting the organ size, maintaining the dynamic balance of cell proliferation, apoptosis and other functions [1]. With the abnormal Hippo pathway, the cells will proliferate excessively or apoptosis insufficiently, and the organ will grow out of control, which will eventually lead to the tumorigenesis and tumour progression [2]. The cores of Hippo pathway consist of the mammalian sterile20-like kinases serine/threonine kinases 1/2 (MST1/2), the large tumour suppressor serine/threonine protein kinases 1/2 (LATS1/2), as well as their scaffold proteins Salvador homologue 1 (SAV1; also called WW45) and Mps one binder kinase activator proteins (MOBs). Mechanistically, MST1/2 phosphorylate and activate LATS1/2 complexed with SAV1 and MOB1 [3,4]. Then, activated LATS1/2 phosphorylate the transcriptional regulators, including yes-associated protein (YAP) and transcriptional co-activators with PDZ-binding motif (TAZ). Phosphorylated YAP/TAZ lose their activation by sequestering in the cytoplasm via interaction with 14-3-3 proteins, then are degraded through the ubiquitin-proteasome pathway [5]. On the other hand, as the transcriptional regulators, YAP/TAZ bind to multiple transcription factors, such as TEADs, Smads, PAXs, TBX5 and RUNX2 [6], and regulate genes involved in stemness, differentiation, proliferation and apoptosis via nuclear translocation.

Besides, the abnormal high expression of YAP/TAZ have been detected in various tumours, such as hepatocellular carcinoma (HCC) [7], breast cancer [8], prostate cancer [9], non-small cell lung cancer [10] and ovarian cancer [11]. An increasing number of studies have confirmed that YAP promotes the tumorigenesis and tumour progression in a various of ways, including promoting cell growth and inhibiting cell apoptosis [12]. One report has described that YAP (not TAZ) could suppress tumour in breast cancer [13]. However, the similar function of TAZ have not been well demonstrated. Allowing for the homology of TAZ with YAP, we hypothesis that TAZ probably get functionality similar to YAP. To assess this issue, we established an inducible expression system of TAZ in T-Rex-293 cells and a stable expression system of TAZ in HEK293 cells. Our study proved that TAZ could act as an oncogene to promote cell proliferation and inhibit cell apoptosis.

## MATERIALS AND METHODS

### Cell culture and reagents

T-Rex-293 cell line was presented by Professor Quan Chen (Chinese Academy of Sciences, Beijing, China). T-Rex-293 cells and HEK293 cells were cultured in RPMI 1640 medium (BIOROC). All mediums were supplemented with 10% FBS and were grown in a humidified environment at 37°C with 5% CO_2_. Doxcycline (Dox) was purchased from Sigma–Aldrich and was prepared as a 2 mg/ml stock solution in sterile ddH_2_O. Giemsa was purchased from Solarbio. Celastrol (purity >98%) was purchased from Mingrui. Stock solutions of Celastrol were prepared in DMSO, stored at −20°C and freshly diluted to the desired concentration before use. The maximal final concentration of DMSO in the culture medium was lower than 0.1%.

The article "TAZ promotes cell growth and inhibits Celastrol-induced cell apoptosis" was published in 2016. Journal: Biosci Rep.

### Plasmid transfection and inducible expression system/stable cell line establishment

To establish the inducible/stable TAZ expression cell line, the open reading frame of human TAZ was cloned into the eukaryotic expression vector pcDNA4/TO/myc-His B (Invitrogen). The primers for TAZ clone are as follows: Forward: 5′-CCCAAGCTTATGAATCCGGCCTCGGCG-3′, Reverse: 5′-CGGAATTCCGGTACAGCCAGGTTAGAAAGGGC-3′. Transfections were performed in 70–80% confluent T-Rex-293 cells and HEK293 cells using LipofectAMINE2000 Reagent (Invitrogen), according to the manufacturer's protocol. Then the cells were selected with 100 μg/ml Zeocin (Invitrogen). The resistant mono-clone was verified by western blot and designated 293-TR/TAZ and HEK293/TAZ, and their corresponding control cells were designated 293-TR/control and HEK293/control.

### Cell growth curve and cell colony formation assay

For the cell growth curve assay, the indicated cells in exponential growth were plated at a density of 50 cells/mm^2^ in triplicate. 293-TR/control and 293-TR/TAZ cells were treated with Dox or not for 7 days, and T-Rrex-293 cells were treated with Celastrol (0.5 μM) or not for 6 days. Cell numbers were counted as indicated with a haematocytometer and an Olympus inverted microscope.

For cell colony formation assay, 293-TR/control and 293-TR/TAZ cells were plated 500 cells/well in six-well plates in triplicate and treated with Dox or not respectively. T-Rex-293 cells with Celastrol (0.5 μM) or not were plated 800 cells/well in six-well plates in triplicate. After approximately 2 weeks, the colonies were washed with PBS, fixed with formaldehyde and stained with Giemsa staining solution. Colonies larger than 100 μm in diameter were counted under an Olympus inverted microscope.

### Tumour xenograft model

Equal numbers (2×10^6^) of HEK293/control and HEK293/TAZ cells were harvested by trypsinization, washed with 1× PBS and resuspended in 0.1 ml of saline. A total number of five (6-week old) female nude mice were given bilateral subcutaneous injections with HEK293/control and HEK293/TAZ cells. The mice were kept in pathogen-free environments and checked every 2 days. The mice were sacrificed 30 days after injection. The weights of the tumour xenografts were measured at the end of the experiment.

The article "TAZ promotes cell growth and inhibits Celastrol-induced cell apoptosis" was published in 2016. Journal: Biosci Rep.

### MTT assay

For dose-dependent and time-dependent proliferation assay, nearly 20000 of T-Rex-293 cells were seeded into 96-well culture plate each well treated with Celastrol at different concentrations (0.25–5 μM). Each concentration was plated in 4 wells, with medium only wells used as the controls. The cells were cultured for 24, 48 and 72 h. Four hours before the end of the incubation, 20 μl MTT (5 mg/ml) were added to each well and 150 μl of DMSO were added to stop the reaction. Viable cell numbers were measured at a wavelength of 570 nm with the Model 680 Microplate Reader (Bio-Rad Laboratories).

### TdT-mediated dUTP Nick end labelling assay

Apoptotic cells were confirmed with the *in situ* cell death detection kit, Alkaline Phosphatase (Roche Applied Science), in accordance with the manufacturer's instructions. T-Rex-293, 293-TR/control and 293-TR/TAZ cells were grown on coverslips. The following process was performed according to the manufacturer's protocol. Cells were mounted cell side downwards on a microscope slide, and the apoptotic cells (brown staining) were counted under a microscope. Three fields were randomly counted for each sample.

### Western blot

Cells were harvested and lysed in RIPA buffer (Cell Signaling Technology), then western blot analysis was performed with the use of conventional protocols as described previously [14]. Total proteins were separated by SDS/PAGE, and transferred on to nitrocellulose membranes. The antibodies were used including β-actin (1:5000, Sigma–Aldrich), PARP (1:1000, Cell Signaling Technology), TAZ (1:1000, Santa Cruz Biotechnology), protein kinase B (Akt; 1:1000, Cell Signaling Technology), pho-Akt (Ser^473^; 1:1000, Cell Signaling Technology), B-cell lymphoma-2 (Bcl-2; 1:1000, Santa Cruz Biotechnology), Bcl-2 associated X protein (Bax; 1:1000, Santa Cruz Biotechnology). After extensively washed, the membranes were incubated with anti-mouse or anti-rabbit IgG-horseradish peroxidase conjugate antibody (Zhongshan Golden Bridge Biotechnology Company) for 1 h at room temperature and developed with a Luminol Chemiluminescence Detection Kit (Zhongshan Golden Bridge Biotechnology Company). Membranes were reprobed for β-actin antibodies for normalization and accurate quantification. Each result for western blot was repeated three times at least.

### Immunohistochemistry

Sections of 5 μm thickness were dewaxed in xylene and rehydrated in serial dilutions of ethanol. Antigen retrieval was carried out in 0.01 M sodium citrate buffer (pH 6.0) for 10 min by microwave oven heating. Then endogenous peroxidase activity was blocked by 3% hydrogen peroxide for 20 min, and nonspecific staining was blocked by 5% BSA for 1 h. The slides were incubated with anti-TAZ (1:100, Santa Cruz Biotechnology) and anti-PCNA (1:1000, Santa Cruz Biotechnology) overnight at 4°C and then incubated with secondary antibody for 30 min, followed by incubation with streptavidin peroxidase for 15 min. 3,3′-Diaminobenzidine tetrachloride (DAB) was applied to identify peroxidase activity. Each incubation step was performed at room temperature and was followed by sequential washed for 3 min each for three times in PBS. Finally, sections were dehydrated in alcohol and cleared in xylene.

The article "TAZ promotes cell growth and inhibits Celastrol-induced cell apoptosis" was published in 2016. Journal: Biosci Rep.

### Quantitative real-time PCR (q-PCR)

Total RNA was extracted with TRIZOL Reagent (Invitrogen), and then reverse-transcribed to cDNA with M-MLV Reverse Transcriptase (Promega). Q-PCR was performed with triplicate samplings of the reverse-transcribed cDNAs on a StepOnePlus Real-Time PCR System (Applied Biosystems) with SYBR Green PCR core reagents (Applied Biosystems), and analysed with StepOne Software. The primers used were as follows:

ANKRD (human):
5′-AGTAGAGGAACTGGTCACTGG-3′/5′-TGGGCTA-GAAGTGTCTTCAGAT-3′;
CYR61 (human):
5′-CCTTGTGGACAGCCAGTGTA-3′/5′-ACTTGGGC-CGGTATTTCTTC-3′;
CTGF (human):
5′-AGGAGTGGGTGTGTGACGA-3′/5′-CCAGGCAGT-TGGCTCTAATC-3′;
GAPDH (human):
5′-CTCCTGCACCACCAACTGCT-3′/5′-GGGCCATC-CACAGTCTTCTG-3′;

### Statistical analysis

The results were expressed as mean±S.D. or ± S.E.M. A Student's two-tailed non-paired *t*-test was used to determine significant differences between treatment and control groups in all experiments. *P*<0.05 was considered statistically significant.

## RESULTS

### TAZ promoted cell growth *in vitro* and *in vivo*

We utilized the T-Rex-293 system to establish an inducible 293-TR/TAZ cell line. As shown in Figure 1(A), only when treated with Dox for 24 h, the exogenous protein level of TAZ increased significantly in 293-TR/TAZ cell line, whereas the expression of TAZ in 293-TR/control cell line (treated with Dox or not) was hardly detected. To better investigate the effect of TAZ on T-Rex-293 cells, cell growth curve and cell colony formation assay were performed. The cell growth curves showed that 293-TR/TAZ cells grew obviously faster when treated with Dox, and the growth rate of the other three groups (293-TR/TAZ cells without Dox and 293-TR/control cells with Dox or not) were nearly the same (Figure 1B). Furthermore, 293-TR/TAZ cells with Dox treatment could form more colonies than the cells without Dox, also than 293-TR/control cells with or without Dox (Figures 1C and 1D). To further address the effect of TAZ *in vivo*, we established a stable expression system of TAZ in HEK293 cells. The resistant mono-clone was designated HEK293/control or HEK293/TAZ. The protein level of TAZ in HEK293/TAZ cells was obviously higher than HEK293/control cells (Figure 1E). The result of tumour xenograft growth in nude mice showed that HEK293/TAZ cells led to larger tumour formation compared with HEK293/control cells (Figures 1F and 1G). As shown in Figure 1(H), tumour analysis showed the protein levels of TAZ and Proliferating Cell Nuclear Antigen (PCNA) were increased in the tumour xenograft of HEK293/TAZ cells, as compared with the control group. All these data indicated that overexpression of TAZ could significantly promote cell growth and proliferation *in vitro* and *in vivo*.

The article "TAZ promotes cell growth and inhibits Celastrol-induced cell apoptosis" was published in 2016. Journal: Biosci Rep.

**Figure 1:** TAZ promoted cell growth *in vitro* and *in vivo* (**A**) The protein levels of TAZ in 293-TR/control and 293-TR/TAZ cells with or without Dox treatment for 24 h were evaluated by western blot. β-Actin was used as a loading control. (**B**) The cell growth curves of 293-TR/control and 293-TR/TAZ cells. Cells were treated with or without Dox, and cell numbers were counted as indicated. Results represent means±S.D. (*n*=3). (**C**) The colony formation of 293-TR/control and 293-TR/TAZ cells. Five hundred cells/well were seeded into six-well plates and treated with Dox or not for 2 weeks. (**D**) The cell colony numbers of 293-TR/control and 293-TR/TAZ cells were analysed. Values are means±S.E.M. (*n*=3). ***P<0.001. (**E**) The protein levels of TAZ in HEK293/control and HEK293/TAZ cells were evaluated by western blot. β-Actin was used as a loading control. (**F**) HEK293/control and HEK293/TAZ cells were injected bilateral subcutaneously into nude mice. The mice were killed 30 days after injection (*n*=5 for each group). (**G**) The weights of tumour xenografts were measured. Results represent means±S.E.M. ***P<0.001. (**H**) The expression of TAZ and PCNA in the tumour xenograft of HEK293/control cells and HEK293/TAZ cells were detected by immunohistochemistry.

### Celastrol suppressed cell growth and induced cell apoptosis in T-Rex-293 cells

Celastrol is derived from the Chinese medicinal plant *Tripterygium wilfordii* [15] and can inhibit cell proliferation [16], induce cell apoptosis [17], suppress invasion/migration [18] and angiogenesis [19]. In our study, T-Rex-293 cells were treated with Celastrol at different concentrations (0.25–5 μM) as indicated for 24, 48 and 72 h respectively. As shown in Figure 2(A), the growth of T-Rex-293 cells was significantly inhibited by Celastrol in a dose- and time-dependent manner. The cell growth curve showed that Celastrol obviously inhibited the growth of T-Rex-293 cells (Figure 2B). Moreover, the colony numbers of T-Rex-293 cells treated with Celastrol was much less than the cells without treatment (Figures 2C and 2D). To further identify whether Celastrol-induced cell growth inhibition was partially due to increased apoptosis, western blot and TdT-mediated dUTP Nick end labelling (TUNEL) assay were performed. As shown in Figure 2(E), the PARP cleavage was definitely observed in T-Rex-293 cells treated with Celastrol compared with the untreated cells. TUNEL assays showed that approximately 87.0% cells were TUNEL-positive in Celastrol treatment group, compared with 3.5% in control group (Figures 2F and 2G). In summary, these data demonstrated that Celastrol inhibited cell growth and induced cell apoptosis in T-Rex-293 cells.

The article "TAZ promotes cell growth and inhibits Celastrol-induced cell apoptosis" was published in 2016. Journal: Biosci Rep.

**Figure 2:** Celastrol suppressed cell growth and induced cell apoptosis in T-Rex-293 cells (**A**) Growth inhibition of T-Rex-293 cells treated with Celastrol at different concentration (0.25–5 μM) and different time-point (24, 48 and 72 h). (**B**) The cell growth curves of T-Rex-293 cells treated with or without Celastrol (0.5 μM 48 h). Cell numbers were counted as indicated. Results represent means±S.D. (*n*=3). (**C**) The colony formation of T-Rex-293 cells treated with or without Celastrol (0.5 μM 48 h). Eight hundred cells/well were seeded into six-well plates for 2 weeks. (**D**) The cell colony numbers of T-Rex-293 cells treated with or without Celastrol (0.5 μM 48 h) were analysed. Values are means±S.E.M. (*n*=3). ***P<0.001. (**E**) Western blot analysis of cleaved PARP in T-Rex-293 cells treated with or without Celastrol (0.5 μM) for 48 h. β-Actin was used as a loading control. (**F**) TUNEL assay was used to detect the apoptotic phenotype induced by Celastrol (0.5 μM 48 h). TUNEL-positive (apoptotic) cells were stained brown (magnification 100×). (**G**) The ratio of apoptosis cells was quantified. Values are means±S.E.M of three measurements in each group. ***P<0.001.

### Overexpression of TAZ could attenuate Celastrol-induced cell apoptosis of T-Rex-293 cells

TAZ is nearly 60% homologous with YAP and YAP could inhibit cell apoptosis [12], so we next determined whether TAZ had the similar function. As Figure 3(A) shown, Dox-induced overexpression of TAZ could inhibit Celastrol-induced PARP cleavage in 293-TR/TAZ cells; When treated with Celastrol (0.5 μM) for 48 h, the percentage of TUNEL-positive cells was obviously reduced from 86.8 to 22.9% in 293-TR/TAZ cells after Dox induction, however, 293-TR/control cells with or without Dox treatment had almost the same ratio of TUNEL-positive cells (Figures 3B and 3C). Our data indicated that overexpression of TAZ could partially inhibit Celastrol-induced cell apoptosis. To investigate the possible mechanism by which TAZ attenuate Celastrol-induced cell apoptosis, we firstly detected the mRNA levels of several TAZ target genes, including ankyrin repeat domain-containing protein (ANKRD), cysteine-rich 61 (CYR61), connective tissue growth factor (CTGF) [20–23]. The results showed that the expressions of ANKRD, CYR61, CTGF were significantly up-regulated in 293-TR/TAZ cells after Dox induction, and were slightly decreased when treated with Celastrol (0.5 μM 48 h; Figure 3D). These data suggested that TAZ may resist cell apoptosis through its target genes. Furthermore, some studies demonstrated that suppression of Akt activation could partially contribute to Celastrol-induced cell apoptosis [24–26]. In the present study, we found Celastrol treatment did not influence the total Akt protein expression, but could decrease the phosphorylation of Akt and Dox-induced overexpression of TAZ increased the phosphorylation of Akt (Figure 3E). Moreover, western blot analysis showed that Celastrol treatment could increase the expression of Bax and decrease the expression of Bcl-2, but induced overexpression of TAZ could attenuate the effect that mentioned above. These data indicated that TAZ may resist Celastrol-induced cell apoptosis through activating phosphatidylinositol 3-kinase (PI3K)/Akt pathway and changing the balance of pro-apoptotic protein Bax and anti-apoptotic protein Bcl-2.

The article "TAZ promotes cell growth and inhibits Celastrol-induced cell apoptosis" was published in 2016. Journal: Biosci Rep.

**Figure 3:** Overexpression of TAZ could attenuate Celastrol-induced apoptosis in T-Rex-293 cells (**A**) Celastrol (0.5 μM) and DMSO were added to 293-TR/control and 293-TR/TAZ cells in the absence and presence of Dox for 48 h. TAZ and cleaved PARP were detected by western blot. β-Actin was used as a loading control. (**B**) Celastrol (0.5 μM) and DMSO were added to 293-TR/control and 293-TR/TAZ cells in the absence and presence of Dox for 48 h respectively. TUNEL assay was used to detect the apoptotic phenotype. TUNEL-positive (apoptotic) cells were stained brown (magnification 100 ×). (**C**) The ratio of apoptotic cells was quantified. Values are means±S.E.M. (*n*=3). ***P<0.001. (**D**) 293-TR/control cells and 293-TR/TAZ cells were treated with Celastrol (0.5 μM) and DMSO in the absence and presence of Dox for 48 h, then the mRNA expression of ANKRD, CYR61 and CTGF were detected by real-time PCR. Values are means±S.E.M. (*n*=3). ***P<0.001. (**E**) 293-TR/control cells and 293-TR/TAZ cells were treated with Celastrol (0.5 μM) and DMSO in the absence and presence of Dox for 48 h, then Akt, pho-Akt (Ser^473^), Bcl-2 and Bax were detected by western blot. β-Actin was used as a loading control.

The article "TAZ promotes cell growth and inhibits Celastrol-induced cell apoptosis" was published in 2016. Journal: Biosci Rep.

## DISCUSSION

Increasing evidence implicates deregulation of Hippo pathway in a variety of cancer. As the major downstream effectors of Hippo pathway, YAP and TAZ are homologous and previous studies demonstrate that most of their biological functions are the same. In the matter of regulating the cell or tissue property, YAP/TAZ play vital roles inapico-basal polarity, mechanotransduction, cell–cell adhesion and contact inhibition [27]. Besides, YAP/TAZ can regulate cell competition, stem cell maintenance, metastasis and regeneration [28]. As oncogenes, both of YAP and TAZ can promote the occurrence and development of tumour.

To date, there has been a considerable body of evidence that links YAP/TAZ to tumorigenicity in cancers. Overexpression of YAP is generally common in a wide variety of tumours, including colon cancer [29], lung cancer [10], gastric cancer [30], liver cancer [31] and breast cancer [8]. YAP can promote cell proliferation, inhibit cell apoptosis, lead to loss of cell contact inhibition and promote cell malignant transformation [32]. Importantly, activation of the LATS kinase results in an increased cytoplasmic phosphorylated YAP accompanied by an induction of apoptosis [33]; when LATS is inhibited, it results in an accumulation of nuclear YAP and then YAP-dependent transcriptional regulation, the consequence of YAP activation can inhibit cell apoptosis [34]. Moreover, the kinases JNKs can phosphorylate YAP to regulate cell apoptosis [35]. Intriguingly, YAP also can accelerate cell apoptosis in the condition of DNA damage. As a transcriptional activated cofactor, YAP can enhance the transcription of the apoptosis-relative genes such as p73 [36] and p53 [37]. YAP promotes apoptosis, which most often occurs in the chemotherapy-induced DNA damage. A previous study reported that phosphorylation of YAP is a crucial regulatory process for its function as a tumour suppressor in certain breast cancers [13]. All these shows that YAP has contradictory roles in cancer progression.

Although YAP and TAZ act as oncogenes, they still have some apparent differences [38]: YAP knockout animals are embryonic lethal [39], but TAZ null mice have renal cysts and lead to end stage kidney disease [40,41]; however, the deletion of both YAP and TAZ causes the exceptionally early death in mice, suggesting there is a potential synergy between YAP and TAZ [42]. Moreover, a study shows that the mRNA expression of TAZ is a prognostic indicator for colon cancer progression, but YAP is not [43].

Compared with TAZ, YAP has more significant effect on cell proliferation and apoptosis [44], but our results indicated that TAZ could also promote cell proliferation. In the present study, we chose T-Rex-293 cell line to construct an inducible expression system of TAZ. In accordance with our expectations, overexpression of TAZ accelerated cell growth *in vitro*. Moreover, the latency of tumour formation in nude mice injected with HEK293/TAZ cells was shorter than the tumours injected with HEK293/control cells (results not shown), which confirmed that TAZ could promote tumour formation *in vivo*. The immunohistochemical results of PCNA further confirmed that TAZ could promote cell proliferation. Furthermore, our cell immunochemistry results proved the same conclusion *in vitro* (results not shown). In addition, previous study demonstrated YAP/TAZ depletion suppress cell growth [32], which is consistent with our study.

The article "TAZ promotes cell growth and inhibits Celastrol-induced cell apoptosis" was published in 2016. Journal: Biosci Rep.

In contrast, TAZ acts as an oncogene to induce epithelial–mesenchymal transition (EMT), and increase cell migration and invasion [45], which is different from YAP. The mutation of TAZ in breast cancer patients with metastases is significantly more than the primary breast cancer patients, which suggests that TAZ may be involved in breast cancer metastasis [46]. Similarly, TAZ can enhance tumour cell metastasis and invasion in the lung cancer, colorectal cancer and glial cell sarcoma. However, there is no direct evidence prompting TAZ can inhibit cell apoptosis. A recent report only indicated that siRNA-mediated knockdown of TAZ could increase apoptosis [47]. Our study further proved that TAZ could have anti-apoptotic ability, which confirmed its oncogenetic roles, but the mechanism of TAZ anti-apoptosis remains to be elucidated.

As we know CYR61 and CTGF are direct target genes of TAZ. Previous studies have demonstrated that CYR61 is a metastatic biomarker and a driver of gastric cardia adenocarcinoma (GCA) [48]. Promotion of angiogenesis and cell proliferation is the major function of CYR61 in tumour progression [49]. CTGF is a matricellular protein which plays an important role in promoting fibrosis and scarring in the skin, kidney, liver, brain and lung [50,51]. Moreover, CTGF may be an adverse prognostic factor in male breast cancer (MBC) [22]. Our results suggested that the anti-apoptotic function of TAZ may be relevant with the up-regulation of CYR61 and CTGF and the decrease in Akt phosphorylation which leads to cell apoptosis [25,26,52,53] may be a mechanism for Celastrol-induced cell apoptosis. On the other hand, some studies indicated that CYR61 and CTGF could increase the phosphorylation of Akt [54–56]. Hence, TAZ may restore Celastrol-induced cell apoptosis by stimulating Akt signalling pathway activation via up-regulation of CYR61 and CTGF.

The article "TAZ promotes cell growth and inhibits Celastrol-induced cell apoptosis" was published in 2016. Journal: Biosci Rep.

The Bcl-2 family containing pro-apoptotic member Bax and anti-apoptotic member Bcl-2, play a pivotal role in the regulation of apoptosis [57]. Our data also showed that Celastrol treatment increased the expression of Bax, decreased the expression of Bcl-2. But overexpression of TAZ could reverse the changes of above-mentioned proteins. It is very likely that the anti-apoptotic potential of TAZ is mediated through suppression of apoptotic gene expression (Bax) and induction of anti-apoptotic gene expression (Bcl-2).

In conclusion, overexpression of TAZ not only could promote cell growth *in vitro* and *in vivo*, it could also inhibit drug-induced apoptosis through the activation of PI3K/Akt signalling pathway and regulation of apoptosis-related proteins (Bax/Bcl-2). Our results reaffirm the oncogenetic role of TAZ and provide clue to improve our understanding of the functions of TAZ in cancers. In view of the above-mentioned roles of TAZ in cell fate determination, it may serve as a novel biomarker for cancers and an effective and selective target for cancer therapy.

## Abbreviations

Akt/PKB: protein kinase B
ANKRD: ankyrin repeat domain-containing protein
Bax: B-cell lymphoma-2 associated X protein
Bcl-2: B-cell lymphoma-2
CTGF: connective tissue growth factor
CYR61: cysteine-rich 61
Dox: doxcycline
LATS1/2: large tumour suppressor serine/threonine protein kinases 1/2
MOB: Mps one binder kinase activator protein
MST1/2: mammalian sterile20-like kinases serine/threonine kinases 1/2
PI3K: phosphatidylinositol 3-kinase
SAV1: also called WW45, Salvador homologue 1
TAZ: transcriptional co-activators with PDZ-binding motif
TUNEL: TdT-mediated dUTP Nick end labelling
YAP: yes-associated protein
